The article "An epithelial–mesenchymal transition-related long noncoding RNA signature correlates with the prognosis and progression in patients with bladder cancer" was published in 2021. Journal: Biosci Rep.

# An epithelial–mesenchymal transition-related long noncoding RNA signature correlates with the prognosis and progression in patients with bladder cancer

**DOI:** 10.1042/BSR20203944

**Published:** 2021-01-05

**Authors:** Hang Tong, Tinghao Li, Shun Gao, Hubin Yin, Honghao Cao, Weiyang He

**Affiliations:** 1 Department of Urology, The First Affiliated Hospital of Chongqing Medical University, Chongqing 400016, China; 2 Central Laboratory, The First Affiliated Hospital of Chongqing Medical University, Chongqing 400016, China; 3 Department of Urology, Mianyang Central Hospital, Mianyang 621000, Sichuan Province, China; 4 Department of Urology, RongChang Traditional Chinese Medicine Hospital, Chongqing 402460, China

**Keywords:** bioinformatic, bladder cancer, epithelial‐mesenchymal transition, lncRNA signature, Prognosis

## Abstract

Bladder cancer is a common malignant tumour worldwide. Epithelial–mesenchymal transition (EMT)-related biomarkers can be used for early diagnosis and prognosis of cancer patients. To explore, accurate prediction models are essential to the diagnosis and treatment for bladder cancer. In the present study, an EMT-related long noncoding RNA (lncRNA) model was developed to predict the prognosis of patients with bladder cancer. Firstly, the EMT-related lncRNAs were identified by Pearson correlation analysis, and a prognostic EMT-related lncRNA signature was constructed through univariate and multivariate Cox regression analyses. Then, the diagnostic efficacy and the clinically predictive capacity of the signature were assessed. Finally, Gene set enrichment analysis (GSEA) and functional enrichment analysis were carried out with bioinformatics. An EMT-related lncRNA signature consisting of TTC28-AS1, LINC02446, AL662844.4, AC105942.1, AL049840.3, SNHG26, USP30-AS1, PSMB8-AS1, AL031775.1, AC073534.1, U62317.2, C5orf56, AJ271736.1, and AL139385.1 was constructed. The diagnostic efficacy of the signature was evaluated by the time-dependent receiver-operating characteristic (ROC) curves, in which all the values of the area under the ROC (AUC) were more than 0.73. A nomogram established by integrating clinical variables and the risk score confirmed that the signature had a good clinically predict capacity. GSEA analysis revealed that some cancer-related and EMT-related pathways were enriched in high-risk groups, while immune-related pathways were enriched in low-risk groups. Functional enrichment analysis showed that EMT was associated with abundant GO terms or signaling pathways. In short, our research showed that the 14 EMT-related lncRNA signature may predict the prognosis and progression of patients with bladder cancer.

## Introduction

Bladder cancer is the most common neoplasm of urological system, and the muscle invasive bladder cancer (MIBC) makes up to approximately 15–25% of new cases. Even the nonmuscle invasive bladder cancer (NMIBC) has approximately 10% probability of progression to MIBC [1,2]. Radical cystectomy is the typical treatment for MIBC; however, approximately 50% of patients have local recurrence and metastasis [3,4]. Accurate diagnosis and detailed classification are crucial to the clinical treatment for bladder cancer [5]. To explore, biomarkers to predict the survival and progression of patients with bladder cancer will be helpful to the diagnosis and treatment.

The article "An epithelial–mesenchymal transition-related long noncoding RNA signature correlates with the prognosis and progression in patients with bladder cancer" was published in 2021. Journal: Biosci Rep.

Epithelial–mesenchymal transition (EMT) is a phenomenon of epithelial cells transforming into mesenchymal cells, which is a process of cell dedifferentiation or redifferentiation [6]. Through the EMT process, the migration and motility of cancer cells are enhanced, contributing to the invasion and metastasis. Epithelial tumours account for more than 95% of the pathological types of bladder cancer [7], so EMT may affect the pathogenesis and progression of bladder cancer. In addition, EMT can also mediate the activation of multiple transcription factors, participate in the repair of cell DNA damage, and promote chemotherapy resistance of tumour cells by enhancing tumour stemness [8]. Hence, it is critical to discover EMT-related biomarkers that can serve as early diagnostic and prognostic biomarkers for patients with bladder cancer.

Bioinformatics can help identify potential biomarkers of prognosis and progression, and in this way to predict survival outcomes in patients with cancer [9,10]. Long noncoding RNAs (lncRNAs) constitute a class of noncoding RNA molecules that regulate the growth of cancer cells and progression [11], and they are potential biomarkers to predict cancer risk and survival outcomes [12]. Therefore, we postulated that EMT-related lncRNAs may be diagnostic and monitoring biomarkers for patients with bladder cancer. In this research, we constructed a prognosis and progression signature based on 14 EMT-related lncRNAs and evaluated its ability to independently and accurately predict the prognosis and progression of patients with bladder cancer.

## Materials and methods

### Data acquisition

The RNAseq expression information and corresponding clinical profiles of patients with bladder cancer were obtained from TCGA database (https://portal.gdc.cancer.gov/). A total of 402 bladder cancer cases were randomly divided into training set (*n*=201) and validation set (*n*=201) by R software using the simple random grouping method (Supplementary File S1). The prediction signature was constructed with training set and verified with the validation set and the whole set (*n*=402). The 200 EMT-related genes (Supplementary File S2) were obtained from gene set ‘Hallmark Epithelial-mesenchymal transition’ in The Molecular Signatures Database (broadinstitute.org/gsea/msigdb).

The article "An epithelial–mesenchymal transition-related long noncoding RNA signature correlates with the prognosis and progression in patients with bladder cancer" was published in 2021. Journal: Biosci Rep.

### Construction of the EMT-related lncRNAs prognostic signature

The Pearson correlation between lncRNAs and EMT-related genes was analyzed. A lncRNA with a correlation coefficient |*R*^2^|>0.4 and *P*<0.05 was considered to be an EMT-related lncRNA (Supplementary File S3). The univariate Cox analysis was used to identify EMT-related lncRNAs whose expression levels were significantly associated (*P*<0.05) with the overall survival (OS) of the patient with bladder cancer. The hazard ratios (HRs) were used to identify risk-related lncRNAs (HR>1) and protective lncRNAs (HR<1). Subsequently, the candidate 38 EMT-related lncRNAs were subjected to multivariate Cox regression analysis to evaluate their contribution as independent prognosis factors in patient survival. Thus, we identified 14 target EMT-related lncRNAs as candidates for the prognosis signature.

### Evaluation of the EMT-related lncRNAs prognostic signature

The risk scores were calculated by the following formula:

$$\text{Risk}\;\text{Score}=\sum_{i=1}^{n}Coef(i)\times x(i),$$

where Coef (i) and *x*(i) represent the estimated regression coefficient and the value of each EMT-related lncRNA expression, respectively. The patients with bladder cancer were grouped into high- and low-risk group according to the median risk score. The OS of patients between the high-risk and low-risk group was compared by the survival curve. The diagnostic efficacy and clinicopathological characteristic of the 14 EMT-related lncRNAs signature were evaluated by the receiver-operating characteristic (ROC) curves. Furthermore, the efficiency of the risk score of our signature to independently predict the survival was assessed by univariate and multivariate Cox regression analyses.

### Establishment the nomogram

We constructed a nomogram by integrating traditional clinical variables and the risk score to analyze the probable 3- and 5-year OS of patients with bladder cancer. Calibration plots and time-dependent ROC curves were analyzed to assess the nomogram.

### Gene set enrichment analysis (GSEA) and functional enrichment analysis

Gene set enrichment analysis (GSEA) was used to analyze significant functional phenotypes in the high-risk group and low-risk group. KEGG gene sets (c2.cp.kegg.v7.2.symbols.gmt) was obtained from the Molecular Signatures Database. After performing 1000 permutation, the enriched gene sets were obtained based on a standard of false discovery rate (FDR) value <0.25 and *P*<0.05. Functional enrichment analysis of GO and KEGG of the mRNA associated with the lncRNA signature were completed using R software (https://www.r-project.org/, version 3.6.2).

The article "An epithelial–mesenchymal transition-related long noncoding RNA signature correlates with the prognosis and progression in patients with bladder cancer" was published in 2021. Journal: Biosci Rep.

### Statistical analysis

The data were processed using the PERL programming language (http://www.perl.org/, Version 5.30.2). Statistical analyses were performed using the GraphPad Prism 8.0 software or the R software in a double-blind manner. *P*<0.05 was regarded as statistically significant.

## Results

### Identification of the signature of 14 EMT-related lncRNAs in patients with bladder cancer

First, we identified 525 EMT-related lncRNAs through Pearson correlation analysis of the lncRNAs from the bladder cancer cases and 200 EMT-related genes, the cutoff values are |*R*^2^|>0.4 and *P*≤0.05. Next, univariable Cox regression analysis between the 525 EMT-related lncRNAs and the survival data showed that 38 lncRNAs were associated with the OS of bladder cancer patients (Supplementary File S4). Then, multivariate Cox regression analysis between the 38 lncRNAs and the survival data found that 14 EMT-related lncRNAs were independent prognostic factors in patients with bladder cancer. Among these lncRNAs, 5 lncRNAs were unfavorable factors (AC105942.1, AL049840.3, SNHG26, C5orf56, AL139385.1) and 9 lncRNAs were confirmed to be favorable prognostic factors for BLCA (TTC28-AS1, LINC02446, AL662844.4, USP30-AS1, PSMB8-AS1, AL031775.1, AC073534.1, U62317.2, and AJ271736.1) (Table 1).

**Table 1:** 14 EMT-related lncRNAs significantly associated with the OS of BLCA patients

Gene symbol	Ensemble ID	Location	*Β* (cox)	HR	*P*
TTC28-AS1	ENSG00000235954	chr22:27,919,368-28,008,581	-0.3367241	0.71410581	0.00187
LINC02446	ENSG00000256039	chr12:10,553,362-10,575,688	-0.0871411	0.91654775	0.00906
AL662844.4	ENSG00000272501	chr6:31,192,361-31,198,037	-0.4306588	0.65008068	0.0036
AC105942.1	ENSG00000235501	chr1:94,927,361-94,963,616	0.05873331	1.06049238	0.0035
AL049840.3	ENSG00000253096	chr14:103,725,728-103,725,825	0.20025402	1.22171306	0.00382
SNHG26	ENSG00000228649	chr7:22,854,126-22,873,537	0.27094356	1.31120106	0.04341
USP30-AS1	ENSG00000256262	chr12:109,051,791-109,054,033	-0.1678379	0.84549087	0.00035
PSMB8-AS1	ENSG00000204261	chr6:32,844,078-32,846,500	-0.0607832	0.94102724	0.00144
AL031775.1	ENSG00000272345	chr6:24,700,907-24,701,793	-0.1808984	0.83452013	0.00015
AC073534.1	ENSG00000268442	chr19:24,162,193-24,163,447	-0.2777473	0.75748824	0.00487
U62317.2	ENSG00000272821	chr22:50,523,926-50,524,780	-0.0400036	0.96078599	0.00604
C5orf56	ENSG00000197536	chr5:132,410,636-132,488,702	0.3825973	1.46608752	0.01303
AJ271736.1	ENSG00000270726	chrX:156,004,218-156,022,236	-0.2025423	0.81665196	0.00649
AL139385.1	ENSG00000275880	chr13:110,613,082-110,616,353	0.20924811	1.23275082	0.01327

The article "An epithelial–mesenchymal transition-related long noncoding RNA signature correlates with the prognosis and progression in patients with bladder cancer" was published in 2021. Journal: Biosci Rep.

### The prognostic impact of 14 EMT-related lncRNA signature

Among the training set, the validation set, and the whole set, the patients with bladder cancer were divided into two groups according to the risk score (Figure 1A). The OS period was longer in the low-risk group than that of the high-risk group (Figure 1B). The diagnostic efficacy of the 14 EMT-related lncRNAs signature was evaluated by the time-dependent ROC curves, in which all the values of the area under the ROC (AUC) were more than 0.73 (Figure 1C). The results above suggested that the 14 EMT-related lncRNAs signature had an excellent capacity of predicting survival period in bladder cancer.

**Figure 1:** The EMT-related lncRNA signature in the training set, the validation set, and the whole set (**A**) Patients sorted by risk score and survival status. (**B**) The survival curve analysis of our EMT-related lncRNA signature. (**C**) Time-dependent ROC curves analysis.

### The 14 EMT-related lncRNA signature was associated with bladder cancer progression

We evaluated the correlation between the risk scores and the clinicopathological features. The results showed no significant correlation between the risk scores and gender of patients (*P*=0.2280). However, patients in >65 years, AJCC stage III-IV, T stage 3-4, N stage 1-3 and M stage1 groups showed significantly higher risk scores compared with patients in ≤65 years (*P*=0.0081), AJCC stage I-II (*P*=0.0001), T stage 1-2 (*P*=0.0006), N stage 0 (*P*=0.0063) and M stage0 (*P*=0.0042) groups, separately (Figure 2A–F). These results suggested that the 14 EMT-related lncRNA signature was associated with bladder cancer progression.

**Figure 2:** The 14 EMT-related lncRNA signature was associated with bladder cancer progression The correlation between the signature risk scores and the clinicopathological features, such as (**A**) Age (>65 vs. ≤65; *P*=0.0081), (**B**) gender (female vs. male; *P*=0.2280), (**C**) AJCC stage (stage I-II vs. stage III-IV; *P*=0.0001), (**D**) T stage (stage 1–2 vs. stage 3–4; *P*=0.0006), (**E**) N stage (stage 0 vs. stage 1–3; *P*=0.0063), (**F**) M stage (stage 0 vs. stage 1; *P*=0.0042).

### The 14 EMT-related lncRNA signature was an independent factor

The prognostic ability of the 14 EMT-related lncRNA signature in bladder cancer was assessed by univariate and multivariate Cox regression analysis. The results showed that the risk score based on our signature was significantly related to the OS of the bladder cancer patients (*P*<0.001) (Figure 3A,B). The ROC curve analysis indicated that the AUC value of the risk score based on our signature was 0.759, which was higher than that of other clinicopathological parameters (Figure 3C). The above results suggested that our EMT-related lncRNA signature was an independent prognostic factor to predict the survival period of patients with bladder cancer.

The article "An epithelial–mesenchymal transition-related long noncoding RNA signature correlates with the prognosis and progression in patients with bladder cancer" was published in 2021. Journal: Biosci Rep.

**Figure 3:** The 14 EMT-related lncRNA signature was an independent factor (**A**) Univariate Cox regression analysis showed the correlation between OS and various clinicopathological parameters and the risk score. (**B**) Multivariate Cox regression analysis showed that the risk score was the independent prognostic indicator for OS. (**C**) ROC curve analysis showed the prognostic accuracy of clinicopathological parameters and the EMT-related lncRNA prognostic risk score.

### Stratification analyses

We performed the stratified analysis of patients with bladder cancer based on clinicopathological information. Compared with the low-risk group, the patients in the high-risk group had shorter OS period in several stratums, such as age > 65 years (*P*<0.001), age ≤ 65 years (*P*<0.001), male (*P*<0.001), female (*P*<0.001), Stage I-II (*P*=0.006), Stage III-IV (*P*<0.001), T1-2 (*P*<0.001), T3-4 (*P*<0.001), N0 (*P*<0.001), N1-3 (*P*<0.001), M0 (*P*<0.001). However, the OS rates between the high-risk and low-risk groups were similar for M1 patients (*P*=0.455; Figure 4), probably because of the smaller sample size. The result showed that our EMT-related lncRNA signature was powerful to predict the survival period of bladder cancer patients in different gradation of age, gender, and AJCC stage.

**Figure 4:** Stratification analyses Survival curve analysis showed the OS rates of the high- and low-risk bladder cancer patients stratified by age, gender, and AJCC stages.

### Establishment of the nomogram

The nomogram can be used to diagnose or predict the onset or progression of a disease [13]. We established a nomogram according to the risk score and other clinicopathological parameters including age, gender, AJCC stage, T stage, and N stage (Figure 5A). The calibration plots worked better than the reference line to predict the 3- and 5-year OS (Figure 5B,C). The AUC of the nomogram at 3- and 5-year were 0.799 and 0.798, respectively, in the ROC curves (Figure 5D).

**Figure 5:** Establishment of the nomogram (**A**) A nomogram by integrating traditional clinical variables and the risk score. (**B** and** C**) The calibration plots for 3- and 5-year OS. (**D**) Time-dependent ROC curves showed that the AUC of the nomogram at 3- and 5-year.

### Gene set enrichment analysis

GSEA results indicated that EMT and cancer-related pathways (renal cell carcinoma, glioma, endometrial cancer, melanoma, focal adhesion, Wnt signaling pathway, and TGF-β signaling pathway) were significantly enriched in the high-risk bladder cancer group (Figure 6A,C). While the immune-related pathways (antigen processing and presentation, primary immunodeficiency, graft versus host disease, autoimmune thyroid disease) were significantly enriched in the low-risk bladder cancer group (Figure 6B,D). These results suggested that a high prognostic signature risk score correlates with EMT and cancer, whereas low prognostic signature risk score correlates with enhanced immune function.

The article "An epithelial–mesenchymal transition-related long noncoding RNA signature correlates with the prognosis and progression in patients with bladder cancer" was published in 2021. Journal: Biosci Rep.

**Figure 6:** GSEA of high- and low-risk patients based on the EMT-related lncRNA prognostic signature (**A** and** C**) GSEA results showed significant enrichment of cancer- and EMT-related signaling pathways in the high-risk BCLA patients. (**B** and** D**) GSEA results showed significant enrichment of immunoregulatory signaling pathways in the low-risk patients.

### Construction of the lncRNA-mRNA co-expression network and functional enrichment analysis

The potential functions of the 14 EMT-related lncRNAs in BLCA were investigated by constructing the lncRNA-mRNA co-expression network using Cytoscape. The lncRNA-mRNA co-expression network contained 82 lncRNA-mRNA pairs based on the threshold parameters (Pearson correlation coefficient |*R*| > 0.4 and *P*<0.05) (Figure 7A). Among the 82 lncRNA-mRNA pairs, 67 mRNAs were significantly correlated with the 14 lncRNAs in the prognostic signature. The Sankey diagram showed the relationship between the 67 mRNAs and 14 lncRNAs (Figure 7B). The top three GO terms for the biological processes were extracellular matrix organization, positive regulation of cell adhesion, and extracellular structure organization. The top three GO terms for the cellular components were collagen-containing extracellular matrix, basement membrane, and cell leading edge. The top three GO terms for molecular functions were extracellular matrix structural constituent, integrin binding, and cell adhesion molecule binding (Figure 7C,D). KEGG pathway analysis confirmed that cytokine–cytokine receptor interaction, focal adhesion, and proteoglycans in cancer were the most significant enriched pathways (Figure 7E,F).

**Figure 7:** The EMT-related lncRNA–mRNA co-expression network and functional enrichment analyses (**A**) Diagrammatic representation of the EMT-related lncRNA–mRNA network. (**B**) The Sankey diagram showed the degree of connection between the mRNAs and EMT-related lncRNAs (risk/protective). (**C** and **D**) GO analysis results. (**E** and** F**) KEGG pathway analysis results.

The article "An epithelial–mesenchymal transition-related long noncoding RNA signature correlates with the prognosis and progression in patients with bladder cancer" was published in 2021. Journal: Biosci Rep.

## Discussion

Bladder cancer is sensitive to neither radiotherapy nor chemotherapy, and is prone to resistance during the treatment. Thanks to the improvement of surgical methods and medical therapy, great progress has been made in the treatment of bladder cancer. However, the relapse and metastasis after operation has not been solved, and the 10-year survival rate is still unsatisfied [14,15].

There are three types of EMT (type 1, 2, and 3) which exert different functions. Type 1 occurs in the embryonic stage and is related to the growth and development of the embryo [16]. Type 2 participates in wound healing, tissue regeneration and organ fibrosis [17]. Type 3 plays a role in tumour invasion and metastasis, which is often related to the poor prognosis of tumour [18]. The reason why EMT is associated with poor prognosis is that EMT enables cancer cells to acquire mobility, invasiveness, and stem cell-like properties. Therefore, EMT-related biomarkers are potential prognosis and progression biomarkers for patients with cancer. Previous studies on the role of specific EMT-related genes in bladder cancer progression found that [19] the EMT signaling pathway was markedly activated during the subtype transition from the nonmuscle invasive bladder cancer (NMIBC) to the muscle invasive bladder cancer (MIBC). Moreover, they developed a tumour-promoting EMT-related gene signature to act as a negative independent prognostic factor.

In the human genome, only less than 1.5% of the DNA sequences can encode proteins, and the remaining approximately 98.5% of the sequences do not encode proteins, which is called noncoding sequences [20]. The higher the degree of evolution, the larger the proportion of noncoding sequences in the genome. This feature suggests that these noncoding sequences may participate in the extremely complex process of life regulation. Among these noncoding sequences, long noncoding RNA (lncRNA) can regulate gene expression and protein activity by affecting chromatin modification and RNA splicing, thus occupying an important position [21,22]. The role of lncRNA in the occurrence, development, prognosis, and chemotherapy resistance of malignant tumours has become a research hotspot. Recent studies reported that an autophagy-related lncRNA signature accurately predicted the prognosis of patients with bladder cancer [23], and an immune-related lncRNA signature could predict survival in hepatocellular carcinoma [24]. With the continuous indepth study on the molecular mechanism of lncRNA in tumour cells, lncRNA is going to provide important information for the diagnosis, targeted therapy and recurrence monitoring of clinical tumour.

The article "An epithelial–mesenchymal transition-related long noncoding RNA signature correlates with the prognosis and progression in patients with bladder cancer" was published in 2021. Journal: Biosci Rep.

In this research, we systematically analyzed the accuracy of EMT-related lncRNAs on prognostic prediction in bladder cancer using bioinformatics and statistical tools. Firstly, we identified 38 EMT-related lncRNAs that were significantly correlated with OS after the univariate Cox regression analysis of the expression of EMT-related lncRNAs in the bladder cancer patient from the TCGA database. Secondly, 14 EMT-related lncRNAs were selected to construct a prognostic signature based on their performance in the multivariate Cox regression analysis. Then, the risk score of each patient with bladder cancer was calculated according to the expression of the 14 EMT-related lncRNAs in the prognostic signature, and the patient was divided into the high-risk or low-risk group based on his/her median risk score. We found that the OS of the patients with bladder cancer was shorter in the high-risk group than that in the low-risk group. What’s more, the ROC curve analysis validated the accuracy of the EMT-related lncRNA prognostic signature in the patients with bladder cancer.

The EMT-related lncRNA prognostic signature is more reliable than the other traditional clinical indicators in prognostic prediction. The nomogram is an effective and reliable clinical tool to predict survival of patients with cancer [25]. Therefore, we developed a robust nomogram consisting of age, gender, AJCC stage, T stage, N stage, and the risk scores (calculated from the EMT-related lncRNA prognostic signature) to improve the prognostic prediction of the patients with bladder cancer. Calibration plots demonstrated that the nomogram predicted 3- and 5-year survival rates was consistent with the actual one. Overall, the 14 EMT-related lncRNA prognostic signature accurately predicted the OS of patients with bladder cancer and exhibited great potential for clinical applications, including individualized prognosis and therapy.

GSEA analysis revealed significant differences in EMT-related signaling pathways between the high-risk group and low-risk group. The immunoregulatory pathways were enriched in the low-risk group, while some cancer- and EMT-related pathways (TGF-β signaling pathway, Wnt signaling pathway) were enriched in the high-risk group. As a multifunctional cytokine, TGF-β participates in numerous cell biological processes and acts on tumour cells by autocrine and paracrine. TGF-β family is closely related to EMT [26]. In tumour progression, TGF-β can activate a series of signaling pathways, including Notch [27], Wnt [28], and Smad [29] signaling pathways, and the cross-talk of these signaling pathways play a synergistic role to start the EMT process. Wnt/β-Catenin pathway is known as a classic Wnt pathway. β-Catenin can combine with the intracellular domain of E-cadherin to form a complex, which can be connected with actin skeleton to mediate cell adhesion and regulate the invasion and metastasis of tumour cells [30,31]. In addition, there is a nonclassical Wnt pathway, in which the Wnt proteins (Wnt5a, Wnt11, and so on) do not produce Wnt signal through the accumulation of β-Catenin in the nucleus. In the nonclassical Wnt pathway, through the action of calmodulin dependent kinase II and the phosphorylation calmodulin sensitive protein and T nuclear factor NF-AT, intracellular Ca^2+^ is increased and protein kinase C is activated to regulate cell adhesion [32]. Moreover, a lncRNA-mRNA co-expression network was established in the present study. Functional enrichment analysis of GO and KEGG showed that EMT was associated with abundant GO terms or signaling pathways. These results support the recognition that EMT is a key regulator in bladder cancer progression.

The article "An epithelial–mesenchymal transition-related long noncoding RNA signature correlates with the prognosis and progression in patients with bladder cancer" was published in 2021. Journal: Biosci Rep.

There are several disadvantages or limitations in our study. Firstly, the bias of the profile analysed in the study couldn’t be ignorant considering the data acquired from public resource. Secondly, we did not perform subtypes of BLCA analysis associated with EMT due to lack of relevant data of subtypes of BLCA in the database. Finally, further investigations involving biochemical experiments such as quantitative real-time PCR, transwell migration/invasion assay and clinical data analyses are required to further confirm our findings.

In conclusion, we first discovered an EMT-related lncRNA prognostic signature which accurately predicted the survival outcomes of patients with bladder cancer. The validity of the prognostic nomogram established by combining the EMT-related lncRNA prognostic signature and other clinicopathological features for accurately predicting the survival period was confirmed. A high prognostic signature risk score correlates with EMT and cancer, whereas low prognostic signature risk score correlates with enhanced immune function. These data provided valuable insights for future investigations into potential individualized treatments for bladder cancer patients belonging to different risk groups.

## Data Availability

All data generated or analyzed during the present study are included in this published article and its Supplementary Material files.

## Abbreviations

AUC: area under the ROC
EMT: epithelial–mesenchymal transition
FDR: false discovery rate
GSEA: gene set enrichment analysis
lncRNA: long noncoding RNA
OS: overall survival
ROC: receiver-operating characteristic

## References

[1] CumberbatchM., JubberI., BlackP.C., EspertoF., FigueroaJ.D., KamatA.M.et al. (2018) Epidemiology of Bladder Cancer: A Systematic Review and Contemporary Update of Risk Factors in 2018. Eur. Urol. 74, 784–795 10.1016/j.eururo.2018.09.00130268659

The article "An epithelial–mesenchymal transition-related long noncoding RNA signature correlates with the prognosis and progression in patients with bladder cancer" was published in 2021. Journal: Biosci Rep.

[2] AntoniS., FerlayJ., SoerjomataramI., ZnaorA., JemalA. and BrayF. (2017) Bladder Cancer Incidence and Mortality: A Global Overview and Recent Trends. Eur. Urol. 71, 96–108 10.1016/j.eururo.2016.06.01027370177

[3] WilliamsS.B., ShanY., Ray-ZackM.D., HudginsH.K., JazzarU., TylerD.S.et al. (2019) Comparison of Costs of Radical Cystectomy vs Trimodal Therapy for Patients With Localized Muscle-Invasive Bladder Cancer. JAMA Surg. 154, e191629 10.1001/jamasurg.2019.162931166593PMC6551585

[4] ZhanY., DuL., WangL., JiangX., ZhangS., LiJ.et al. (2018) Expression signatures of exosomal long non-coding RNAs in urine serve as novel non-invasive biomarkers for diagnosis and recurrence prediction of bladder cancer. Mol. Cancer 17, 142 10.1186/s12943-018-0893-y30268126PMC6162963

[5] KamounA., de ReynièsA., AlloryY., SjödahlG., RobertsonA.G., SeilerR.et al. (2020) A Consensus Molecular Classification of Muscle-invasive Bladder Cancer. Eur. Urol. 77, 420–433 10.1016/j.eururo.2019.09.00631563503PMC7690647

[6] BakirB., ChiarellaA.M., PitarresiJ.R. and RustgiA.K. (2020) EMT, MET, Plasticity, and Tumor Metastasis. Trends Cell Biol. 30, 764–776 10.1016/j.tcb.2020.07.00332800658PMC7647095

[7] GargM. (2015) Urothelial cancer stem cells and epithelial plasticity: current concepts and therapeutic implications in bladder cancer. Cancer Metastasis Rev. 34, 691–701 10.1007/s10555-015-9589-626328525

[8] AshrafizadehM., ZarrabiA., HushmandiK., KalantariM., MohammadinejadR., JavaheriT.et al. (2020) Association of the Epithelial-Mesenchymal Transition (EMT) with Cisplatin Resistance. Int. J. Mol. Sci. 21, 4002 10.3390/ijms2111400232503307PMC7312011

[9] TianX., XuW., WangY., AnwaierA., WangH., WanF.et al. (2020) Identification of tumor-infiltrating immune cells and prognostic validation of tumor-infiltrating mast cells in adrenocortical carcinoma: results from bioinformatics and real-world data. Oncoimmunology 9, 1784529 10.1080/2162402X.2020.178452932923148PMC7458645

[10] YangJ.L., WangC., CaiJ.H., ChouC.Y., LinY.C. and HungC.C. (2020) Identification of GSN and LAMC2 as Key Prognostic Genes of Bladder Cancer by Integrated Bioinformatics Analysis. Cancers (Basel) 12, 1809, 10.3390/cancers12071809PMC740875932640634

[11] ArunG., DiermeierS.D. and SpectorD.L. (2018) Therapeutic Targeting of Long Non-Coding RNAs in Cancer. Trends Mol. Med. 24, 257–277 10.1016/j.molmed.2018.01.00129449148PMC5840027

[12] WuB., WangK., FeiJ., BaoY., WangX., SongZ.et al. (2018) Novel three-lncRNA signature predicts survival in patients with pancreatic cancer. Oncol. Rep. 40, 3427–3437 3054269410.3892/or.2018.6761PMC6196600

The article "An epithelial–mesenchymal transition-related long noncoding RNA signature correlates with the prognosis and progression in patients with bladder cancer" was published in 2021. Journal: Biosci Rep.

[13] ZhangC., GouX., HeW., YangH. and YinH. (2020) A glycolysis-based 4-mRNA signature correlates with the prognosis and cell cycle process in patients with bladder cancer. Cancer Cell Int. 20, 177 10.1186/s12935-020-01255-232467671PMC7238531

[14] AlmassiN., ChaE.K., VertosickE.A., HuangC., WongN., DasonS.et al. (2020) Trends in Management and Outcomes among Patients with Urothelial Carcinoma Undergoing Radical Cystectomy from 1995 to 2015: The Memorial Sloan Kettering Experience. J. Urol. 204, 677–684 10.1097/JU.000000000000107132294398PMC7483392

[15] HusseinA.A., ElsayedA.S., AldhaamN.A., JingZ., OseiJ., KaoukJ.et al. (2019) Ten-Year Oncologic Outcomes Following Robot-Assisted Radical Cystectomy: Results from the International Robotic Cystectomy Consortium. J. Urol. 202, 927–935 10.1097/JU.000000000000038631188729

[16] WangX., De GeyterC., JiaZ., PengY. and ZhangH. (2020) HECTD1 regulates the expression of SNAIL: Implications for epithelial-mesenchymal transition. Int. J. Oncol. 56, 1186–1198 3231957610.3892/ijo.2020.5002PMC7115742

[17] ForteE., ChimentiI., RosaP., AngeliniF., PaganoF., CalogeroA.et al. (2017) EMT/MET at the Crossroad of Stemness, Regeneration and Oncogenesis: The Ying-Yang Equilibrium Recapitulated in Cell Spheroids. Cancers (Basel) 9, 98 10.3390/cancers908009828758926PMC5575601

[18] ZhangH., HanX., WeiB., FangJ., HouX., LanT.et al. (2019) RSPO2 enhances cell invasion and migration via the WNT/β-catenin pathway in human gastric cancer. J. Cell. Biochem. 120, 5813–5824 10.1002/jcb.2786730362605

[19] CaoR., YuanL., MaB., WangG., QiuW. and TianY., 2020) An EMT-related gene signature for the prognosis of human bladder cancer. J. Cell. Mol. Med. 24, 605–617 10.1111/jcmm.1476731657881PMC6933372

[20] WangJ., ZhuS., MengN., HeY., LuR. and YanG.R. (2019) ncRNA-Encoded Peptides or Proteins and Cancer. Mol. Ther. 27, 1718–1725 10.1016/j.ymthe.2019.09.00131526596PMC6822234

[21] BarthD.A., JuracekJ., SlabyO., PichlerM. and CalinG.A. 2020) lncRNA and Mechanisms of Drug Resistance in Cancers of the Genitourinary System. Cancers (Basel) 12, 214810.3390/cancers12082148PMC746378532756406

[22] LiF., GuoH., LiuB., LiuN., XuZ., WangY.et al. (2020) Explore prognostic biomarker of bladder cancer based on competing endogenous network. Biosci. Rep. 40, BSR20202463 10.1042/BSR2020246333169791PMC7711062

[23] SunZ., JingC., XiaoC. and LiT. (2020) An autophagy-related long non-coding RNA prognostic signature accurately predicts survival outcomes in bladder urothelial carcinoma patients. Aging (Albany NY) 12, 15624–15637 10.18632/aging.10371832805727PMC7467376

The article "An epithelial–mesenchymal transition-related long noncoding RNA signature correlates with the prognosis and progression in patients with bladder cancer" was published in 2021. Journal: Biosci Rep.

[24] ZhangY., ZhangL., XuY., WuX., ZhouY. and MoJ. (2020) Immune-related long noncoding RNA signature for predicting survival and immune checkpoint blockade in hepatocellular carcinoma. J. Cell. Physiol. 235, 9304–9316 10.1002/jcp.2973032330311

[25] MirM.C., MarchioniM., ZargarH., Zargar-ShoshtariK., FaireyA.S., MertensL.S.et al. (2020) Nomogram Predicting Bladder Cancer-specific Mortality After Neoadjuvant Chemotherapy and Radical Cystectomy for Muscle-invasive Bladder Cancer: Results of an International Consortium. Eur. Urol. Focus 10.1016/j.euf.2020.07.00232771446

[26] PallaschF.B. and SchumacherU. (2020) Angiotensin Inhibition, TGF-β and EMT in Cancer. Cancers (Basel) 12, 2785 10.3390/cancers12102785PMC760146532998363

[27] ZhangT.H., LiangL.Z., LiuX.L., WuJ.N., SuK., ChenJ.Y.et al. (2019) LncRNA UCA1/miR-124 axis modulates TGFβ1-induced epithelial-mesenchymal transition and invasion of tongue cancer cells through JAG1/Notch signaling. J. Cell. Biochem. 120, 10495–10504 10.1002/jcb.2833430635938

[28] PelulloM., ZemaS., NardozzaF., ChecquoloS., ScrepantiI. and BellaviaD. (2019) Wnt, Notch, and TGF-β Pathways Impinge on Hedgehog Signaling Complexity: An Open Window on Cancer. Front. Genet. 10, 711 10.3389/fgene.2019.0071131552081PMC6736567

[29] TongH., YinH., HossainM.A., WangY., WuF., DongX.et al. (2019) Starvation-induced autophagy promotes the invasion and migration of human bladder cancer cells via TGF-β1/Smad3-mediated epithelial-mesenchymal transition activation. J. Cell. Biochem. 120, 5118–5127 10.1002/jcb.2778830320898

[30] KatohM. (2018) Multi-layered prevention and treatment of chronic inflammation, organ fibrosis and cancer associated with canonical WNT/β-catenin signaling activation (Review). Int. J. Mol. Med. 42, 713–725 2978611010.3892/ijmm.2018.3689PMC6034925

[31] RöperJ.C., MitrossilisD., StirnemannG., WaharteF., BritoI., Fernandez-SanchezM.E.et al. (2018) The major β-catenin/E-cadherin junctional binding site is a primary molecular mechano-transductor of differentiation in vivo. Elife 7, e33381 10.7554/eLife.3338130024850PMC6053302

[32] MaL. and WangH.Y. (2007) Mitogen-activated protein kinase p38 regulates the Wnt/cyclic GMP/Ca2+ non-canonical pathway. J. Biol. Chem. 282, 28980–28990 10.1074/jbc.M70284020017684012

